The article "Riluzole Stimulates BDNF Release from Human Platelets" was published in 2015. Journal: Biomed Res Int.

# Riluzole Stimulates BDNF Release from Human Platelets

**DOI:** 10.1155/2015/189307

**Published:** 2015-01-06

**Authors:** Patrick Türck, Marcos Emílio Frizzo

**Affiliations:** Department of Morphological Sciences, Institute of Basic Health Sciences, Federal University of Rio Grande do Sul, Rua Sarmento Leite, 500, 90050-170 Porto Alegre, RS, Brazil

## Abstract

Brain-derived neurotrophic factor (BDNF) has several functions in the central nervous system, where it contributes to brain development and its functionality through affecting neuronal survival and activity and also modulating neurotransmitter levels. This neurotrophin is also found in the serum, but its origin and peripheral function remain unknown. Although the source of circulating BDNF is uncertain, it is stored in platelets and can be released through pharmacological treatment. Decreased levels of BDNF in the serum have been related to the pathophysiology of depression, and this relationship is reinforced by the reversal of this condition by treatment with antidepressants. Recently, riluzole has been proposed for the treatment of depression because it has the ability to lower extracellular glutamate levels and increase BDNF expression; and both mechanisms could be associated with its antidepressant action. Considering that riluzole enhances BDNF levels in the serum of patients, we investigated if treatment with this drug could stimulate the release of this neurotrophin from human platelets obtained from healthy subjects. When platelets were incubated with riluzole for 4 h, the basal value of BDNF (92.9 ± 11.1 pg 10^−6^ platelets) was significantly increased (P < 0.05, n = 27). This stimulatory effect was achieved at low concentrations of riluzole (from 10 *µ*M) and was not observed when platelets were incubated with the drug for 24 h. The direct action of riluzole evoking BDNF release from human platelets at therapeutic concentrations is important and may contribute to the understanding of its mechanisms of action in the treatment of depression.

## 1. Introduction

Brain-derived neurotrophic factor (BDNF) contributes to brain development [1, 2] and is related to neuronal survival and activity since it acts as a modulator of neurotransmitter levels and participates in neuronal plasticity [3, 4]. In the human, monkey, and rat, BDNF is also found in the serum at significant levels [5–7], but the origin and function of this neurotrophin remain unknown. Investigators have mentioned the brain as the source for this circulating neurotrophin [8], even though it has been demonstrated that BDNF crosses the blood-brain barrier (BBB) in both directions [9, 10]. Indeed, BDNF may originate from neurons and glia cells [9, 10]; however, it is also released at significant rates by other peripheral tissues, such as different epithelia, where its amounts may reach levels higher than those found in the central nervous system (CNS) [11]. Other examples of BDNF origins other than from CNS are white cells [12–14] and platelets; the latter contain significant quantities of this protein and might provide an important source of this circulating neurotrophin [5]. It has been shown that more than 99% of blood BDNF proteins are stored in platelets and that these proteins can be released into the serum [6] through pharmacological treatment [15, 16].

The article "Riluzole Stimulates BDNF Release from Human Platelets" was published in 2015. Journal: Biomed Res Int.

Recent studies have reported changes in serum BDNF levels in patients with psychiatric diseases [17–20], such as major depressive disorders [21]. The relationship between decreased BDNF levels and the pathophysiology of depression is supported by several reports [21–25]. Pandey et al. [26] showed that gene expression of BDNF in lymphocytes and its protein expression in platelets from adult and pediatric depressed patients were significantly decreased, and the authors proposed that it could be a target for antidepressant drugs. In fact, some antidepressants increase BDNF expression [27] and also may evoke BDNF release from platelets, in a dose-dependent manner after direct treatment* in vitro* [15]. The BDNF concentration in the serum increases after intravenous treatment with an antidepressant, and the effect of these drugs on BDNF release from platelets was related to the level of this neurotrophin in the peripheral blood [15].

Recently, glutamatergic modulators have been proposed as a strategy for the treatment of mood disorders [28]. Among the drugs proposed is riluzole (2-amino-6-trifluoromethoxy benzothiazole), which was originally developed as an anticonvulsant [29] but has been used in a number of trials for psychiatric conditions in which glutamate excess has been proposed as part of the pathologic mechanism [30–33]. Different mechanisms of action have been reported for riluzole [32], which probably explains its complex pharmacological effects. For instance, a stimulatory effect on glutamate uptake was observed at low glutamate concentration [34], and this ability to lower extracellular glutamate levels was suggested as its mechanism of antidepressant action, at least partially [32]. However, other mechanisms cannot be ruled out, since riluzole also increases the BDNF expression [35, 36], which could also contribute to its antidepressant action [32]. Treatment with riluzole significantly increases serum levels of BDNF in patients [37]. Considering that BDNF in the blood is thought to originate from platelets and is evoked by antidepressant drugs, we decided to investigate if riluzole could stimulate the release of this neurotrophin from human platelets.

The article "Riluzole Stimulates BDNF Release from Human Platelets" was published in 2015. Journal: Biomed Res Int.

## 2. Methods

### 2.1. Subjects

Human blood was collected from 27 healthy male volunteers registered as donors in the Hemotherapy Service of the Clinical Hospital of Porto Alegre, Rio Grande do Sul, Brazil. The study was carried out in accordance with The Code of Ethics of the World Medical Association (Declaration of Helsinki) for experiments involving humans. Informed consent was obtained from the donors and their privacy rights were observed.

### 2.2. Procedures

Two samples of 4 mL were taken from the antecubital vein of each donor and placed in vacutainers (BD Franklin Lakes, USA) containing K_3_-EDTA. Immediately, they were gently inverted 10 times and placed in an ABX Micros ES 60 hematology analyzer (HORIBA ABX SAS, Japan) to determine the number of platelets in each blood sample. Platelets were isolated as previously described by Mangano and Schwarcz [38]. The vacutainers were then centrifuged at 300 ×g for 5 min at 4°C and the platelet-rich plasma (PRP) was obtained. The supernatant (PRP) was carefully removed with a plastic pipette tip, with care not to disturb the leukocyte layer. The volume of PRP collected from each sample was recorded and the PRP was transferred to a microcentrifuge tube. The PRP was then centrifuged at 7000 ×g for 10 min at 4°C. The plasma was discarded and the pellet was resuspended in 0.5 mL of 0.32 M phosphate-buffered sucrose (pH 7.4 at 4°C). The suspension, hereafter referred to as the platelet concentrate (PC), was repeatedly passed through a plastic pipette tip of 1 mL until the visible platelet aggregates were eliminated. An additional 0.5 mL of buffered sucrose was added to the suspension and the solution was mixed with 5 gentle inversions. The PC was again centrifuged at 7000 ×g for 5 min at 4°C. The supernatant was discarded, and the pellet was resuspended in a volume of 0.32 M phosphate-buffered sucrose (pH 7.4 at 4°C), equal to one-fifth of the initial volume of PRP obtained. After that, the two PC suspensions obtained from each subject were blended and the number of platelets was determined again. As previously observed by our group, the platelets should be counted in the PC, after the platelets are washed [39]. The mean platelet volume (MPV) and platelet distribution width (PDW) were also determined in both the whole blood and the PC to evaluate potential variations in the platelets during the processing. The incubation was performed in a 96-well plate; to each well were added 20 × 10^6^ platelets in 130 *μ*L of Tris-citrate buffer (112.8 mM NaCl, 4.5 mM KCl, 1.1 mM KH_2_PO_4_, 1.1 mM MgSO_4_, 11 mM Na_3_-citrate, 25 mM Tris-HCl, and 10.2 mM glucose), pH 6.5. Drugs were diluted in Tris-citrate buffer, and the final volume in the well was 150 *μ*L.

The article "Riluzole Stimulates BDNF Release from Human Platelets" was published in 2015. Journal: Biomed Res Int.

### 2.3. BDNF Protein Assay

BDNF levels in the supernatants were measured using a ChemiKine Brain Derived Neurotrophic Factor Sandwich ELISA kit (Millipore, USA) following the manufacturer's instructions. All BDNF measurements were performed in triplicate on 96-well plates, and a standard curve was calculated for each experiment. Samples from the supernatants were diluted 1 : 16 in phosphate buffer solution (pH 7.4) for BDNF measurement. The platelet BDNF content was calculated by dividing the result for BDNF obtained by the total platelet count from the same individual and was expressed as pg BDNF 10^−6^ platelets. The optical density of each well was measured using a microplate reader (EZ Read 400, Biochrom, UK) set to 450 nm; the optical densitometry data were analyzed with the software Galapagos (Biochrom, UK). The sensitivity was 7.8 pg BDNF mL^−1^ and the assay exhibited no cross-reactivity with other members of the nerve growth factor family.

### 2.4. MTT Assay

The MTT assay was utilized to determine the effect of riluzole or sertraline on platelet viability after 4 or 24 h of drug exposure. For shorter incubation times (4 h), 20 *μ*L MTT (5 mg mL^−1^) was added to each well at the time that the platelets were plated, and it was maintained at room temperature by 4 h. For longer incubation times (24 h), 20 *μ*L MTT (5 mg mL^−1^) was added to each well 20 h after plating and maintained at room temperature for an additional 4 h. Subsequently, 150 *μ*L of DMSO was added to dissolve the formazan, which was detected using a microplate reader (EZ Read 400, Biochrom, UK). The absorption was read at 570 nm; the value obtained (UAbs) was expressed as UAbs 20 · 10^−6^ platelets.

### 2.5. Statistical Methods

Values are reported as mean ± SEM, and the statistical analysis was conducted using SPSS. The data were normally distributed, as determined by the Shapiro-Wilk normality test, and were analyzed through one-way ANOVA (for BDNF) or two-way ANOVA (for MTT) followed by Tukey's multiple comparisons test (alpha at 0.05).

## 3. Results

We used washed platelets to test if riluzole could stimulate BDNF release, acting directly on these cells. Initially, the platelet indices (cell count, MPV, and PDW) were measured in whole blood and again after obtaining the PC, to evaluate if these parameters changed during the processing. Then, the platelet number quantified in each PC was used to normalize the BDNF quantity in the respective experiment. Our data showed that the platelet count should be determined after the PC is obtained, since the cell number was reduced during the process (yield of 42 ± 8%). Analysis of PC showed an absence of contaminant cells; and despite the loss of platelets, the MPV and PDW indices were not changed after the cells were obtained. The platelet indices MPV and PDW in the whole blood were 8.1 ± 0.6 *μ*m^3^ and 14.9 ± 1.0%, respectively. When compared with PC, we did not observe significant differences for MPV and PDW, which showed levels of 8.2 ± 0.6 *μ*m^3^ and 15.5 ± 1.2%, respectively. In our analysis, the platelet number achieved in the PC was 1545 ± 338 × 10^3^ mm^−3^.

The article "Riluzole Stimulates BDNF Release from Human Platelets" was published in 2015. Journal: Biomed Res Int.

In our experimental conditions, the basal values of BDNF released from platelets of donors ranged from 9.0 to 220.2 pg 10^−6^ platelets. The wide distribution of BDNF quantified in the study group is depicted in Figure 1.

Given the recent evidence that riluzole treatment causes a significant increase of BDNF in the serum of patients [37], the effect of this drug on BDNF release from human platelets was tested. Platelets from healthy volunteers were treated with different concentrations of riluzole for 4 or 24 h at room temperature. When platelets were incubated with riluzole for 4 h, the basal value of BDNF as quantified from the controls (92.9 ± 11.1 pg 10^−6^ platelets) was significantly increased (*P* < 0.05). Even for platelets from donors who showed lower basal levels of BDNF, treatment with riluzole stimulated the release of this neurotrophin. The increase mediated by riluzole was significant beginning with 10 *μ*M (15%) and was maintained up to 40 *μ*M (22%) and 100 *μ*M (20%). We also tested the effect of 1 *μ*M riluzole, which did not differ from the control (Figure 2).

The effect of riluzole on the BDNF release determined in our model was reproducible in repeated runs, even though it varied from individual to individual. Considering this variability in the basal levels of BDNF among different donors (Figure 1), in each set of experiments, the drug effect was compared with the respective control. We also used sertraline (0.3 *μ*M) as a positive control, since it was recently reported to be a potent inducer of BDNF release from platelets [15]. However, contrary to expectations, in our experiments, the sertraline did not significantly stimulate BDNF release (data not shown).

The increase in the release of BDNF evoked by riluzole was not observed when platelets were incubated with the drug for 24 h. In order to determine if platelet viability was affected by riluzole during the exposure, we used the MTT assay. Hence, the activity of NAD(P)H-dependent cellular oxidoreductase enzymes was evaluated after 4 and 24 h incubation. The viability of the untreated platelets did not differ after the two incubation periods, although slightly less formazan was produced after 24 h (Figure 3).

The article "Riluzole Stimulates BDNF Release from Human Platelets" was published in 2015. Journal: Biomed Res Int.

## 4. Discussion

We evaluated the platelet parameters MPV and PDW, since these indices have been reported to correlate with platelet function [40]. MPV is a measurement that is commonly used to describe platelet size and is an indicator of activated platelets [41, 42], while PDW represents the range of variability in platelet volume [43]. Taking into account that MPV and PDW did not change before the platelets were obtained and after they were processed, we can state that the platelets used in this study were not activated at the time of exposure to riluzole. Importantly, we did not select a subpopulation of these cells, since no significant difference was observed in the PDW. Another important point is that our protocol used only platelets, and, consequently, the BDNF quantified cannot be attributed to contaminant cells such as leukocytes.

In our study, we observed a direct action of riluzole, evoking BDNF release from human platelets. The stimulatory effect was achieved at low concentrations (from 10 *μ*M), which could be important information for the clinical use of riluzole. Although this increase was not as large as found for another antidepressant [15], the stimulatory effect was reproducible when compared with the respective controls, despite the variations among different donors. The absence of a sertraline effect on BDNF release might be due to our use of human cells, whereas Watanabe et al. [15] used rat platelets. Unfortunately, Watanabe and coauthors did not report the basal values of BDNF that they obtained, which would allow comparison with our data.

Riluzole evoked an acute effect on the platelets, which was not observed after longer incubation times. The release of BDNF in response to riluzole acutely (4 h) and not later (24 h) suggests that its effect derived from evoking neurotrophin release from the platelet pool and is not related to a stimulatory effect on neurotrophin synthesis. This is in accordance with data showing that mRNA expression of BDNF in human platelets is extremely low [5, 10].

The novel finding that riluzole elicits BDNF release from human platelets is important, since this situation may occur peripherally and also in deep regions of the CNS, where platelets and astrocytes are very close and where this neurotrophin is able to pass through the BBB. Beyond the peripheral consequences of this release mediated by riluzole, the effects of this neurotrophin on the CNS may be complex and significant, especially regarding the glutamatergic system. It has been shown that BDNF exerts acute effects on glutamatergic synaptic transmission and plasticity, that is, enhancing excitatory synaptic transmission through pre- and postsynaptic mechanisms [44]. On the other hand, its stimulatory effect on the expression of astroglial glutamate transporters and the consequent increase in glutamate uptake capacity has also been described [45]. More recently, it was demonstrated that BDNF upregulates the protein expression of the vesicular glutamate transporters (VGLUT1 and VGLUT2) in hippocampal neurons [46], which reinforces the participation of BDNF as a modulator of the glutamatergic synapse.

The article "Riluzole Stimulates BDNF Release from Human Platelets" was published in 2015. Journal: Biomed Res Int.

Clinically, riluzole has been used in trials for psychiatric conditions where glutamate excess is proposed as part of the pathologic mechanism [47]. It is also suggested that it produces antidepressant and anxiolytic effects in the treatment of resistant depression [32]. Its effect in these conditions is associated with the ability to reduce extracellular glutamate levels and also may involve its stimulatory action on BDNF expression [32]. Therefore, the demonstration that riluzole causes BDNF release at low concentrations is significant* in vivo* and shows the importance of studying platelets from patients treated with this drug. Studies to clarify the mechanisms related to BDNF release in human platelets are currently in progress in our laboratory.

## 5. Conclusions

The new effect described for riluzole may contribute to the understanding of the mechanisms involved with its therapeutic action, reinforcing the suggestion for its use in psychiatry, such as in the treatment of depression.

## Figures and Tables

**Figure 1:** Scatter plot of BDNF released from human platelets. The mean of BDNF values (92.9 ± 11.1 pg 10^−6^ platelets) is indicated by the dotted bar (*n* = 27).

**Figure 2:** Stimulatory effect of riluzole on BDNF release. Platelets obtained from healthy donors were incubated with different concentrations of riluzole (1, 10, 40, or 100 μM) for 4 h. Control is represented by the dotted line. Data are presented as mean ± SEM. ^*^Different from control (*n* = 27, *P* < 0.05).

**Figure 3:** Platelet viability during the incubation period. The effect of different concentrations of riluzole on platelet viability was determined at 4 or 24 h of incubation. No significant differences were observed among the groups. Data are presented as mean ± SEM (*n* = 27).
